# Detection of immunological treatment failure among HIV infected patients in Ethiopia: a retrospective cohort study

**DOI:** 10.1186/s12865-015-0120-1

**Published:** 2015-09-16

**Authors:** Wondu Teshome, Ambachew Tefera

**Affiliations:** School of Public and Environmental Health, Hawassa University, Hawassa, Ethiopia; International Center for AIDS Care and Treatment Program (ICAP), Federal Ministry of Health, Addis Ababa, Ethiopia

**Keywords:** HIV type 1, ART, Immunological treatment failure, Ethiopia, Treatment switching

## Abstract

**Background:**

Timely detection of treatment failure with subsequent switch to second-line regimen reduces mortality among HIV infected people on antiretroviral therapy (ART). This paper aims to investigate the detection of immunological treatment failure and switch rate to second line regimen in Ethiopia.

**Methods:**

A retrospective cohort study was conducted among HIV infected patients (age > 15 years) who initiated ART between 2007 and 2009. The required data were collected from patient registers and formats. Data were entered and validated using EpiData software and then exported to SPSS version 20.0 for analysis. Odds ratio with 95 % CI was used to assess whether immunological treatment failure was associated with experiencing unfavorable treatment outcomes (death or lost to follow up).

**Results:**

Records of 293 patients were reviewed with a total of 1545 Person-Years of Observation (PYO). The median baseline CD4 count was 115 cells/mm^3^ (IQR: 64–176). A total of 46 (15.7 %) patients experienced immunological treatment failure. The immunological failure rate was 3.0 per 100 PYO. Treatment was switched to second-line regimen for six (2.1 %) patients. The rate of treatment switch to second-line regimen for any purpose was 0.4 per 100 PYO. Out of the six patients, only two fulfilled the WHO criteria for immunological failure; the remaining four patients had their treatment switched to second-line regimen for other purposes. This implies that only 4.3 % (2/46) of patients with immunological failure were switched to second-line regimen. The risk of experiencing unfavorable outcome was 5.75 (95 % CI 1.11, 29.8) times higher among those who had immunological failure than their counterparts after adjusting for baseline CD4 count.

**Conclusions:**

Majority of patients with immunological treatment failures were not detected and continued taking the failed regimen. Further studies are required to assess and explore why patients with immunological failure are not switched to second-line regimen as per the standard protocol.

## Background

Approximately 35.0 million people were living with HIV in the world by the end of 2013. In the same year, 12.9 million people living with HIV were receiving antiretroviral therapy (ART) globally, out of which 11.7 million were in low and middle-income countries representing 36 % of the 32.6 million people living with the virus in low and middle-income countries [1].

As the ART uptake increases, the emergence of resistant viruses resulting in treatment failure is inevitable and should be anticipated proactively. As a result patients need to be switched to second-line regimen in order to have a sustained viral suppression [1–3].

The diagnosis of treatment failure is guided by viral load testing in high income countries; however, this is not the case in most low income countries because viral load testing is costly and requires advanced infrastructures [2, 3]. Cognizant of this, WHO has designed relatively simple criteria to diagnose treatment failure using immunological and clinical criteria. The definitions of immunological failure are either fall of CD4 count to baseline (or below) or 50 % fall from on-treatment peak value or persistent CD4 levels below 100 cells/mm^3^ [3].

Even though the immunological criteria to diagnose treatment failure was documented to have low positive predictive value and low sensitivity, the extent to which it is being utilized in health facilities has not been well studied in Ethiopia. Thus, in this study we aim to investigate the rate of immunological failure, its detection and switch rate to second-line regimen.

## Methods

### Study setting

The study was conducted in Federal Police Referral Hospital (FPRH). ART program was launched in the hospital in parallel with other public health facilities. FPRH started to provide ART service in 2005. The hospital also provides HIV prevention, care and support services.

### Treatment initiation, eligibility criteria and service delivery model

The ART guideline in Ethiopia is based on the 2008 WHO recommendations. However, there were technical updates as an addendum to the national ART guideline at different times based on the 2010 and 2013 WHO recommendations [4].

According to the national ART guideline, eligibility for initiation of ART is determined using CD4 count and WHO clinical stage. When CD4 count is not available, patients with WHO clinical stage III and IV conditions are eligible for treatment. In addition, patients with WHO clinical stage II conditions with Total Lymphocyte Count (TLC) less than 1,200 cells/ml are considered for treatment [4].

Whereas in the presence of CD4 count, WHO clinical stage III patients with CD4 cell count less than 350 cells/mm^3^ and all patients with WHO clinical stage IV conditions are eligible for treatment. In addition, patients with WHO clinical stage I and II with CD4 cell count below 200 cells/mm^3^ are eligible for treatment [4]. There was no major change in eligibility criteria until 2013 which is beyond the period for cohort selection for this study.

In FPRH, the HIV chronic care services are delivered by trained nurses and health officers. Physicians are available for consultation in case of complications and for patients with advanced disease.

### Study design, study population and sampling procedure

This study was a retrospective cohort study of HIV-infected patients who started ART at the FPRH. The intended service users in FPRH include active and retired police members, their dependents, civilian workers and other civilian residents in the surrounding area.

The current study included patients (age > 15 years) who started ART between January 2007 and December 2009, had follow up in the facility for at least 24 months and had at least four CD4 measurements including the baseline measurement. Transfer-in cases were also included in the study provided that they fulfilled all the other inclusion criteria. The primary end-point was immunological failure using the WHO definitions as outlined above.

In the present study, baseline CD4 count was a measurement occurring closest to the date of starting ART, within a window of 6 months prior to the start of ART to 1 week after ART initiation.

### Data collection procedure

A structured data abstraction format was used to collect the data from patients’ cards and registers. The format was developed using the standardized patient monitoring formats and registers. Patient intake form, follow up card and ART registers as well as the electronic information database were used as data sources. Other clinical charts including laboratory test results were also used to collect the CD4 cell counts.

Unique ART number and the new Health Management Information System (HMIS) card number were used to identify individual patient cards or their data in the electronic database. Socio-demographic characteristics, baseline and follow up clinical and laboratory data, and treatment outcomes were collected from patient cards.

Two data clerks and one case manager (adherence supporter) from FPRH were trained and hired as data collectors. The federal police health service directorate data manager was hired as data collection supervisor. All completed formats were examined for clarity and consistency by the supervisor and finally by the researchers. The data were collected in June /2014.

### Data management and analysis

Data were entered, and validated using EpiData software version 3.1. Each format was given a unique identification number for data entry. A cleaned and compiled data were exported for analysis to SPSS version 20. Proportions, means, medians with measures of dispersion were calculated as deemed necessary. Odds ratios with 95 % CIs were used to assess whether immunological treatment failure was associated with experiencing unfavorable treatment outcomes (death or loss to follow up). For statistical tests, level of significance was set at type-I error of 0.05.

### Ethical considerations

Ethical clearance was obtained from Addis Continental Institute of Public Health and Mekele University joint Institutional Review Board. Permission was obtained from Federal Police Health Service Directorate and FPRH administration. In Ethiopia, patients are not requested for consent to use an already existing data within health facilities. All the information obtained during the course of the study was held in a confidential manner. The data were kept in a locked cupboard. Patient names were not recorded or linked to the results of the study.

## Result

### Selected charts for review

Within the period of interest, there were a total of 741 patients who initiated ART in the hospital. However, only 293 charts fulfilled the inclusion criteria and were included for data abstraction. Figure 1 depicts the result of the patient card selection using flow chart.

**Fig. 1:** Selection steps for the analyzed charts in Federal Police Referral Hospital for patients who initiated ART between January 2007 and December 2009

### Baseline characteristics of the study cohort

Records of 293 patients were reviewed with a total of 1545 Person-Years of Observation (PYO). All the study cohorts initiated treatment between January 2007 and November 2009. Most (58.4 %) of the study cohorts started ART in the month of knowing their HIV infection status. At baseline, the mean age was 36.7 years (SD = 8.6 years) and 64.2 % were males while the sex of 0.7 % were not recorded. The median baseline CD4 count was 115cells/mm^3^ (IQR: 64–176). Majority (75.8 %) of the patients had baseline CD4 count less than 200cells/mm3. In relative terms, the common regimen was D4T/3TC/NVP accounting for 39.2 %. Treatment was switched to second-line regimen for 2.1 % of the cases. Substitution to different drugs within first line regimen was observed for 30.7 % of the cases. Similar results for other variables and disaggregated by immunological failure status is shown in Table 1.

**Table 1:** Baseline characteristics of the study cohort

Variable		Immunologic treatment failure		Total (%)
		Yes (%)	No (%)	
Sex	Male	32 (17.0)	156 (83.0)	188 (64.2)
	Female	14 (13.6)	89 (86.4)	103 (35.2)
	NR	1 (50.0)	1(50.0)	2 (0.7)
Age (In years), at Month0	Mean, SD	34.6, 7.5	36.6, 8.5	36.7, 8.6
	15–34	23 (18.1)	104 (81.9)	127 (43.5)
	35–44	16 (13.3)	104 (86.7)	120 (41.1)
	> = 45	6 (13.3)	39 (86.7)	45 (15.4)
Original First Line Regimen	D4T/3TC/NVP	15 (13.0)	100 (87.0)	115 (39.2)
	D4T/3TC/EFV	59 (78.7)	16 (21.3)	75 (25.6)
	AZT/3TC/NVP	32 (78.0)	9 (22.0)	41 (14.0)
	AZT/3TC/EFV	54 (91.5)	5 (8.5)	59 (20.1)
	TDF/3TC/EFV	2 (66.7)	1 (33.3)	3 (1.0)
Original Regimen substituted	Yes	34 (16.8)	168 (83.2)	202 (68.9)
	No	79 (87.8)	11 (12.2)	90 (30.7)
	NR	0	1	1 (0.3)
Switch to second line regimen	Yes	2 (33.3)	4 (66.7)	6 (2.0)
	No	44 (15.3)	243 (84.7)	287 (98.0)
Baseline CD4 count, cells/mm^3^	Median, IQR	122 (67–190)	114 (63–176)	115 (64–176)
	0–49	6 (12.8)	41 (87.2)	47 (16.2)
	50–99	12 (16.0)	63 (84.0)	75 (25.9)
	100–149	9 (14.3)	54 (85.7)	63 (21.7)
	150–199	8 (12.9)	54 (87.1)	62 (21.4)
	> = 200	10 (23.3)	33 (76.7)	43 (14.8)
Base line functional status	Work	29 (15.9)	153 (84.1)	182 (62.1)
	Ambulatory	9 (15.5)	49 (84.5)	58 (19.8)
	Bedridden	3 (12.0)	22 (88.0)	25 (8.5)
	NR	5 (17.9)	23 (82.1)	28 (9.6)
Body Mass Index. Kg/m2	<18.5	12 (18.8)	52 (81.2)	64 (21.8)
	> = 18.5	15 (13.9)	93 (86.1)	108 (36.9)
	NR	19 (15.7)	102 (84.3)	121 (41.3)
Gap between testing and treatment initiation	Same month	29 (17.0)	142 (83.0)	171 (59.0)
	1–24 months	13 (13.4)	84 (86.6)	97 (33.4)
	>24 months	4 (18.2)	18 (81.8)	22 (7.6)
Adherence	Good	35 (15.2)	195 (84.8)	230 (78.5)
	Fair/ poor	10 (18.5)	44 (81.5)	54 (18.4)
	NR	1 (11.1)	8 (88.9)	9 (3.1)

*NR* Not Recorded, *IQR* Interquartile Range, *SD* Standard Deviation

### Cohort period and treatment outcome

The median retrospective follow up period was 70 months (IQR: 54–76 months). By the time the data collection terminated, 81.2 % were actively on treatment, 4.1 % were lost or dropped from care, 2.0 % died and the rest 12.6 % were transferred out to another facility.

A total of 46 (15.7 %) patients experienced immunological treatment failure. This translates to immunological failure rate of 3.0 per 100 PYO. Out of these 46 patients with immunological failure, the reasons for the failure were drop by more than 50 % of the pick value attained in 45.3 % of the cases, persistently below 100 cells/mm3 after taking ART for at least 24 weeks in 13.3 % of the cases and CD4 count below the baseline value in another 45.3 % of the cases.

Treatment was switched to second-line regimen for six (2.1 %) patients. The rate of treatment switch to second-line regimen for any purpose was 0.4 per 100 PYO. Out of the six patients only two fulfilled the WHO criteria for immunological failure; the remaining four patients had their treatment switched to second-line regimen for other purposes such as regimen simplification. This implies that only 4.3 % (2/46) of immunologically failed patients were switched to second-line regimen.

### Effect of immunological treatment failure on treatment outcome

Next we examined if immunological treatment failure was associated with final follow up status. Accordingly, we found that the proportion of patients experiencing unfavorable treatment outcome was higher among patients with immunological treatment failure than their counterparts. For instance, the proportion of those who died was 6.5 % among patients who had immunological failure whereas it was 1.2 % among the other group (Fig. 2).

**Fig. 2:** Proportion of different follow up outcomes based on experience of immunological treatment failure

When the outcome was dichotomized by taking dead and lost to follow up or drop as unfavorable outcome and the rest as favorable outcome, it was found that the risk of experiencing unfavorable outcome was 4.99 (95 % CI 1.85, 13.44) times higher among those experiencing immunological failure than their counterparts and it became 5.75 (95 % CI 1.11, 29.8) times higher when adjusted for baseline CD4 count.

## Discussion

In the present study, it was found that after a median follow up duration of 70 months (IQR: 54–76 months), 15.7 % of the cohorts experienced immunological failure. The failure rate of 3.0 per 100 PYO observed in our study was slightly less than a study conducted in Haiti which reported failure rate of 4.8 per 100 PYO [5]. This could be because the Haiti study used both clinical and immunological criteria to define treatment failure.

The overall switch rate to second-line regimen of 2.1 % in the current study is very low when compared with other studies from resource-constrained settings [5–10]. These studies reported that majority of the treatment switch to second-line regimen was due to treatment failure and not for treatment simplification [6–10].

The collaborative analysis of data from Zambia and Malawi documented the overall switch rate of 13.4 % among patients with immunological failure [11]; however, in our study only 4.3 % (2/46) of such patients were switched to second-line regimen. This indicates that majority of patients with immunological failure weren’t recognized and switched to second-line regimen in this setting. A similar finding was documented by Keiser et al. who argued that many patients who meet criteria for treatment failure do not switch to second-line regimen resulting in preventable deaths in Sub-Saharan Africa countries [12].

In this study, around 96 % (44/46) of patients with immunological failure continued to take the already failed first-line regimen. This finding was significantly different from the report from Haiti where the health care systems detected 40 % and subsequently switched treatment to second-line regimen [5]. This indicates presence of a big gap in the quality of care being given as a large proportion of treatment failures weren’t detected timely. Despite the low positive predictive value and low sensitivity of the immunological criteria to detect virologic failure [13, 14], failure of the health system to detect and switch treatment to second-line regimen for such patients will worsen the final outcome of HIV patients with immunological failure.

In the current study, we noted that the risk of unfavorable outcome was significantly higher among immunologically failed group. As this is a facility based document review study, we couldn’t further verify the outcomes of those who were lost from care. In order to control for this, if we make the assumption that all patients who were lost from care are alive, the risk of dying remains significantly higher though the confidence interval becomes wide owing to the sample size (OR 5.67, 95 % CI, 1.11, 29.04). Previous studies conducted in Malawi to verify the true outcome of lost patients indicated that around half of such patients were found to be dead and remained undocumented by the health system [15, 16].Other studies previously conducted in similar contexts documented higher death rate among the immunologically failed group who weren’t switched to second-line treatment [17, 18]. Timely switch to second-line regimen was also documented to have a good viral suppression success rate [6] and also to reduce mortality [12].

Diagnosis of treatment failure and timely regimen switch to second-line may also act as a positive push factor for prevention of circulation of resistant viruses in the community. A study conducted by Reynolds et al. found that patients with immunological failure exhibit several types of mutations [19]. The continuation of a failing regimen was also documented to result in rapid accumulations of drug resistance [20]. The circulation of such resistant viruses can have a negative impact on treatment choice, as future patients may present with an already resistant virus which implies that a structured approach for treatment won’t be effective and initial treatment choice will be based on resistance testing [21] which is a very expensive approach in resource-limited settings.

Finally, the study may have limitations which could affect generalization for the whole population on treatment. In the first place many patients were excluded from the cohort because their charts weren’t accessible and/or they didn’t fulfill the inclusion criteria of having at least four CD4 count measurements Kiraga et al. [22] in a recent study have documented that ignoring such outcomes could even over estimate the success of the treatment programs.

## Conclusion

In the current study, it was observed that majority of patients with immunological treatment failures were not detected and such patients continued to take the failed regimen. The proportion of unfavorable outcome was higher among the immunologically failed group. Further studies are required to assess and explore why patients with immunological treatment failure are not switched to second-line regimen as per the standard protocol.

## Availability of data and materials

Not applicable.
